The article "MRF-IUNet: A Multiresolution Fusion Brain Tumor Segmentation Network Based on Improved Inception U-Net" was published in 2022. Journal: Comput Math Methods Med.

# MRF-IUNet: A Multiresolution Fusion Brain Tumor Segmentation Network Based on Improved Inception U-Net

**DOI:** 10.1155/2022/6305748

**Published:** 2022-08-04

**Authors:** Yongchao Jiang, Mingquan Ye, Peipei Wang, Daobin Huang, Xiaojie Lu

**Affiliations:** ^1^School of Medical Information, Wannan Medical College, Wuhu 241002, China; ^2^Research Center of Health Big Data Mining and Applications, Wannan Medical College, Wuhu 241002, China

## Abstract

The automatic segmentation method of MRI brain tumors uses computer technology to segment and label tumor areas and normal tissues, which plays an important role in assisting doctors in the clinical diagnosis and treatment of brain tumors. This paper proposed a multiresolution fusion MRI brain tumor segmentation algorithm based on improved inception U-Net named MRF-IUNet (multiresolution fusion inception U-Net). By replacing the original convolution modules in U-Net with the inception modules, the width and depth of the network are increased. The inception module connects convolution kernels of different sizes in parallel to obtain receptive fields of different sizes, which can extract features of different scales. In order to reduce the loss of detailed information during the downsampling process, atrous convolutions are introduced in the inception module to expand the receptive field. The multiresolution feature fusion modules are connected between the encoder and decoder of the proposed network to fuse the semantic features learned by the deeper layers and the spatial detail features learned by the early layers, which improves the recognition and segmentation of local detail features by the network and effectively improves the segmentation accuracy. The experimental results on the BraTS (the Multimodal Brain Tumor Segmentation Challenge) dataset show that the Dice similarity coefficient (DSC) obtained by the method in this paper is 0.94 for the enhanced tumor area, 0.83 for the whole tumor area, and 0.93 for the tumor core area. The segmentation accuracy has been improved.

## 1. Introduction

Glioma is the most common primary central nervous system tumor and has a high fatality rate. Therefore, gliomas are the key objects of brain tumor segmentation. According to the degree of tumor malignancy, it can be divided into high-grade glioma (HGG) and low-grade glioma (LGG) [1]. The growth rate of LGG is slow, and the patients have better survival prognosis. HGG patients have high mortality and poor survival prognosis. Magnetic resonance imaging (MRI) is an important auxiliary technology in the diagnosis and treatment of brain tumors. It can provide brain images with high soft tissue contrast, no bone artifacts, and no damage [2]. Brain tumor MRI has a variety of sequences, including T1-weighted (T1), contrast enhanced T1-weighted (T1c), T2-weighted (T2), and fluid attenuated inversion recovery (FLAIR) [3]. Doctors often combine multiple MRI sequences to obtain more detailed and comprehensive information about brain tumors.

With the rapid development of deep learning technology, the method based on deep learning has made remarkable achievements in the field of computer vision, and it is also widely used in the field of semantic segmentation of medical images [4]. The structure of brain tissue is very complex, the boundaries of brain tumors are fuzzy, and the size, shape, and location of tumors are very different [5]. These factors increase the complexity and difficulty of brain tumor segmentation. The multilayer network structures such as convolution layer, pool layer, and full connection layer in convolution neural network (CNN) can learn and extract the multilevel features of brain tumor images and can achieve pixel-level classification of brain tumor images [6]. Compared with manual segmentation and traditional segmentation methods, the brain tumor segmentation algorithm based on CNN has higher efficiency and segmentation accuracy [7]. In 2015, Long et al. [8] changed the original full connection layers of CNN into convolution layer and proposed the full connection network (FCN), a pixel level image semantic segmentation network. FCN restores the reduced feature maps to the original image size by upsampling, thereby achieving end-to-end image segmentation. Ronneberger et al. [9] proposed the architecture U-Net for biomedical images, which consists of a contracting path to capture context information and an expansive path to enable accurate localization, and the corresponding feature maps of the contraction path and the expansion path are fused through skip connections. U-Net has achieved good results in the field of medical image segmentation, but the original U-Net is relatively simple, and the network layers are not deep enough, which cannot achieve more accurate results when dealing with the complex brain tumor segmentation task [10]. However, if the depth of the network is increased directly by simple stacking, a large number of parameters will be added, and the network is prone to overfitting and gradient disappearance. At the same time, the continuous downsampling operations in the U-Net reduce the feature resolution, and some of the detailed information is lost, resulting in inaccurate segmentation results [11].

In order to improve network performance, it is necessary to increase the depth of the network, but to avoid the problems of parameter redundancy and gradient disappearance. The inception modules were adopted in the GoogLeNet [12], which also makes GoogLeNet achieve the best performance in the ImageNet Large-Scale Visual Recognition Challenge 2014 (ILSVRC14). The inception module connects the pooling layer and multiple convolution kernels in parallel to construct a dense component to approximate the optimal local sparse structure. Inception modules increase the width of the network, improves the utilization of computing resources within the network, and improves network performance. DeepLab [13] uses atrous convolutions in the network. It can expand the receptive field without adding additional parameters, which can reduce the downsampling operators and prevent the loss of detailed information. At the same time, ASPP module is proposed in DeepLab [14]. ASPP module parallelizes atrous convolutions with different rates, which can integrate the features of objects at different scales. Many studies have shown that the early convolution layers can extract more spatial context information like edges, corners, and textures, which is conducive to the fine segmentation and location of the target. Deeper layers extract more abstract semantic features, which are of great significance for target object recognition, but lack strong spatial information [8, 15]. In U-Net, the corresponding resolution features of the encoder and the decoder are stitched together through skip connections, which can retain the spatial context information of the low-level layers. In this paper, we propose an encoder-decoder architecture based on U-Net, which fuses the multiresolution features of the network to better combine the spatial context features and the abstract semantic features [16]. More details are as follows:

1. We replace the original convolution modules in U-Net with inception modules, which can increase both the depth and width of the network [17]. The parallel structure of the convolution kernels of the inception module makes it have different receptive fields and can better capture multiscale features
2. The continuous downsampling operation reduces the feature resolution and also leads to the loss of image details, so we add atrous convolutions to the model, which can expand the receptive fields without downscaling the image, and will not add extra parameters
3. The spatial detail features extracted by the low-level layers play an important role in the fine segmentation of the image. In this paper, the features with different resolutions in the encoder are upsampled to obtain the same resolution, and then, these feature maps are spliced and finally fused with the corresponding feature maps in the decoder

## 2. Related Work

In recent years, the methods based on CNNs have made significant progress in image semantic segmentation. There are many excellent network architectures with their own characteristics [18, 19]. Full convolution network- (FCN-) based methods can realize pixel-level classification of images and are widely used in the field of image segmentation.

The encoder-decoder structure is a commonly used network structure in image semantic segmentation, which can accept input images of any size and can achieve end-to-end semantic segmentation [20]. U-Net is a commonly used encoder-decoder architecture; it has a relatively simple architecture and is very suitable for medical image segmentation. The encoder of U-Net gradually reduces the feature resolution and increases the receptive field through downsampling, to further extract high-level semantic information. The decoder recovers the spatial context information and achieve precise localization through upsampling operators, which combines the high-resolution features from the contracting path. Some researchers have introduced residual connections [21] and dense connections in the ResNet [22] and DenseNet [23] into U-Net and constructed improved network architectures ResUNet and DenseUNet [24, 25], which have improved segmentation accuracy compared with U-Net. In addition, the attention mechanism is introduced into U-Net to form the Attention U-Net. Before the corresponding features of the encoder are combined with the upsampled output, an attention module is added to readjust the weight of different features, so that the segmentation target can obtain greater attention weight, which is helpful to improve the segmentation accuracy [26].

In the convolutional neural network, the feature resolution is reduced by the downsampling operation, and part of the detailed information will be lost in the process. Yu and Koltun proposed DeepLab network, which enlarges the receptive field and captures multiscale contextual information by atrous convolution with different rates [27]. The atrous space pyramid pooling module (ASPP) is also used in the DeepLab network to capture multiscale features by paralleling multiple atrous convolutions with different rates. However, when the dilation rate of the atrous convolution gradually increases, the proportion of effective feature weights in the atrous convolution will decrease. Therefore, in the DeepLabv3 [28], an improved ASPP module is proposed. By adding global pooling, global information was integrated to obtain better segmentation results. DeepLabv3+ [29] uses an encoding-decoding architecture, the encoder can obtain rich semantic information, and the decoder restores fine object information and uses deep separable convolution, which effectively reduces the number of parameters. In order to improve the network performance, it usually chooses to increase the depth and complexity of the network, but simply deepening the network will increase the number of parameters, which will not only increase the amount of calculation but also easily lead to over fitting. Szegedy et al. [30] proposed the inception module, which clusters the sparse matrix into dense matrix to approximate the optimal local sparse structure, which can effectively improve the computational performance. The parallel structure of convolutions with different sizes can also better capture multiscale features.

## 3. Methods

### 3.1. Inception Module

The network used in this paper is an encoder-decoder architecture based on U-Net. Generally, the first way to improve the network performance is to build a deeper network, but simply increasing the depth of the network will bring a large number of parameters, which will easily lead to over fitting, and the deepening of the network layers will also increase the computational complexity. In order to solve this problem, we need to make the neural network structure sparse, but the computational efficiency of computer processing nonuniform sparse data is low. Therefore, it is necessary to design a module that can not only improve the computational performance but also make the network structure sparse. The structure of inception module is to approximate the optimal local sparse structure by clustering the sparse matrix into dense submatrices. Therefore, this paper uses the inception modules instead of the original convolution modules. The structure of the inception module is a parallel connection of multiple convolution kernels of different sizes, which is more conducive to capturing multiscale features. The inception module has three branches in parallel, one of which is 1 × 1 convolution, and the other two branches are a 3 × 3 convolution and two stacked 3 × 3 convolutions. In order to reduce the number of parameters, the 1 × 1 convolution is used to reduce the number of feature channels, and a BN layer is added after each convolution kernel. To speed up network training and prevent vanishing gradients, a residual connection is added to the inception module [31]. The U-Net uses downsampling to reduce the resolution of the feature maps four times, which can increase the receptive field without using a larger convolution kernel. However, in the process of downsampling and upsampling, part of the detailed information of the image will be lost. Therefore, in order to reduce the downsampling operation, prevent the loss of image detail information, and ensure that sufficient global context information can be obtained, the last downsampling of the encoder is rounded off in the proposed network in this paper, and two inception modules fused with atrous convolutions (A-inception module) are used to obtain different receptive fields by changing the dilation rates of atrous convolutions. The specific module structure is shown in Figures 1 and 2.

### 3.2. Multiresolution Fusion Module

In the original U-Net, the feature maps of the encoder are cropped and fused with the feature maps of the decoder, so that some image detail features can be recovered in the upsampling process. In order to obtain more accurate segmentation, it is necessary to make full use of the spatial detail information. In this paper, a multiresolution feature fusion module (MRF) is constructed between encoder and decoder, which uses richer spatial context information for accurate feature location in the upsampling stage. The module upsamples the low-resolution feature maps in the encoder to obtain the same resolution and then splits these feature maps together. The splicing feature maps are combined with the corresponding feature maps of the decoder through a 3 × 3 convolution. The specific structure is shown in Figure 3.

### 3.3. Network Structure

This paper builds an improved brain tumor segmentation architecture named MRF-IUNet. This architecture uses five inception modules in the encoding stage, each module has three different branches in parallel, and multiple branches have different sizes of receptive fields, which can capture multiscale features. For brain tumor images with large differences in tumor size, obtaining multiscale features is beneficial to improve the segmentation performance and the robustness of network. At the same time, a residual connection is added to each inception module, which is more conducive to the training and convergence of the network. The first three inception modules of the encoder use standard convolution with convolution kernels of 1 × 1 and 3 × 3. The A-inception block1 and A-inception block2 use a 1 × 1 convolution kernel and 3 × 3 atrous convolutions with different dilation rates. The specific structure is shown in Figure 4. The dilation rates rate1, rate2, and rate3 in A-inception block1 and A-inception block2 are 2, 2, 4 and 4, 4, 8, respectively, by increasing the dilation rate of atrous convolution, a larger receptive field can be obtained, which is conducive to obtaining more global context information. In the encoding stage, three downsampling modules are used, and each downsampling module uses 2 × 2 max pooling with stride 2 and the 3 × 3 convolution with stride 2 and splices the outputs of the two as the downsampling output.

The decoding stage also uses five inception modules to form a symmetrical structure with the encoder. The first two modules use A-inception modules that incorporate atrous convolutions, named A-inception block3 and A-inception block4. The dilation rates of the atrous convolutions used are 2, 2, 4 and 4, 4. 8. The latter three inception modules use standard convolutions with convolution kernel of 3 × 3 and 1 × 1. In the decoding stage, the feature map needs to be gradually restored to the same size as the original input image. This architecture uses an upsampling method of bilinear interpolation.

The encoder and decoder are connected by the ASPP module. According to the atrous space pyramid module proposed in DeepLabv3, a 1 × 1 convolution and three 3 × 3 atrous convolutions are connected in parallel, the batch normalization layer (BN) [32] is added after the convolution layer. Global pooling is added to integrate more global context information. The ASPP module connected multiple atrous convolutions with different rates in parallel, thus obtaining receptive fields of different sizes, which can extract more multiscale features. In the [28], when output − stride = 16 (output-stride is the ratio of the scale of the input image to the output feature map), the dilation rates of the three atrous convolutions used by ASPP are 6, 12, and 18, respectively. In this paper, output − stride = 8; through experimental comparison, when the dilation rates are 12, 18, 24, respectively, the segmentation performance of the network is the best. The specific ASPP module structure is shown in Figure 5.

The loss function used in this paper is a linear combination of the cross entropy loss function and the Dice loss function, which can alleviate the problem caused by the imbalance of the samples. The cross entropy loss function and Dice loss function are defined as follows:

(1) $$\begin{array}{c} {\text{Loss}}_{\text{BCE}}=-\frac{1}{N}\overset{N}{\underset{i}{\sum }}\left[y_{i}∙\log\left(p_{i}\right)+\left(1-y_{i}\right)∙\log\left(1-p_{i}\right)\right],\\ {\text{Loss}}_{\text{Dice}}=1-\frac{2\times \sum_{i}^{N}p_{i}y_{i}}{\sum_{i}^{N}p_{i}+\sum_{i}^{N}y_{i}}. \end{array}$$

Calculate the set *N* of all samples, where *y*_*i*_ is the hot coding (0 or 1) of the *i*th sample label, and *p*_*i*_ is the predicted probability of the *i*th sample label.

In this paper, the adaptive moment estimation (Adam) [33] algorithm is used as the gradient optimization algorithm in the back propagation process. The Adam algorithm is an exponentially weighted moving average of small batch stochastic gradients based on the RMSProp algorithm. The advantages of Adam algorithm are simple implementation, high computational efficiency, and low memory requirements, and it is suitable for large-scale data and parameter optimization problems.

## 4. Experimental Results and Analysis

In this paper, we used the Pytorch framework to build the brain tumor segmentation network models. The experimental environment is Intel Xeon Silver 4116 CPU@ 2.10GHz, GPU NVIDIA GeForce RTX2080Ti. 20% of the data in the training set needs to be used as a validation set for initial evaluation of model performance and tuning of hyperparameters, and the rest is used for model training. The hyperparameters batch size, learning rate, and momentum of experimental training are set to 16, 0.0003, and 0.9, respectively.

### 4.1. Experimental Data and Preprocessing

The experimental data used in this paper is the BraTS dataset. BraTS 2018 training dataset is used as the training dataset for this experiment, including the data of 210 HGG patients and 75 LGG patients. Each case contains four MRI sequence images of T1, T2, T1C, and FLAIR and ground truth. The test dataset of the experiment uses the BraTS 2019 training dataset. The original size of each modal MR image is 240 mm × 240 mm × 155 mm. The ground truth segmentation labels are tumor segmentation regions manually annotated by multiple experts, including four types of labels: normal tissue (label 0), necrosis and nonenhancing tumor (label 1), edema (label 2), and enhancing tumor (label 4).

Because the distribution of MRI brain tumor image data is quite different, and the uneven distribution of data will increase the difficulty of network training, which is not conducive to the model learning the distribution rules between different tumor categories, therefore, it is necessary to standardize the image to limit the intensity distribution of the image to a certain range [34]. Since the background information in the original image occupies a large proportion, the problem of data imbalance will occur, so it is necessary to crop the redundant background of the image. Slice the cropped three-dimensional image to obtain two-dimensional image data with the size of 160 × 160. The training dataset needs to discard the slices without lesions to alleviate the category imbalance and combine the slices of each MRI sequence into 4-channel samples as input.

### 4.2. Evaluation Indicators

In order to objectively evaluate the effect and feasibility of the segmentation algorithm, it is necessary to use evaluation indicators to quantify the prediction results. The intersection of union (IOU), dice similarity coefficient (DSC) and positive predictive value (PPV) are used to evaluate the segmentation performance of the model [35]. IOU represents the overlap rate between the predicted value and the ground truth, and the DSC represents the similarity between the predicted value and the ground truth. They are commonly used evaluation indicators in the medical image segmentation. Their expressions are as follows:

(2) $$\begin{array}{c} \text{IOU}=\frac{\text{TP}}{\text{FP}+\text{TP}+\text{FN}},\\ \text{DSC}=\frac{2\text{TP}}{\text{FP}+2\text{TP}+\text{FN}}. \end{array}$$

PPV represents the proportion of true positive samples among all samples predicted to be positive samples by the experiment. The calculation method is as follows:

(3) $$\begin{array}{c} \text{PPV}=\frac{\text{TP}}{\text{TP}+\text{FP}}, \end{array}$$

where TP, FP, and FN represent true positive, false positive, and false negative, respectively. TP represents the correctly segmented positive samples, FP represents the incorrectly segmented negative samples, and FN represents the incorrectly segmented positive samples. The value range of the evaluation indicator is 0-1. The closer the value is to 1, the better the segmentation result.

### 4.3. Experimental Results

In this paper, a multiresolution fusion brain tumor segmentation model based on U-Net is proposed, and the BraTS dataset is used as the experimental dataset. The segmentation areas of brain tumors include whole tumor area (WT), tumor core area (TC), and enhancing tumor area (ET). WT includes enhancing tumor, necrosis, and edema area, and TC includes enhancing tumor area and necrosis; ET only includes enhancing tumor area [36].

Use the training dataset to train the built model, and then, use the test dataset for segmentation test. In order to compare the segmentation effect between the proposed method (MRF-IUNet) and other advanced methods, we selected U-Net, ResUNet, DenseUNet, and Deeplabv3+ for comparison and used the same dataset and parameters to train and test these networks. The segmentation results of each network and the ground truth (GT) are shown in Figure 6. U-Net, ResUNet, DenseUNet, and the proposed method adopt the basic structure of U-Net and use skip connections between the encoder and the decoder, so that the details of segmentation target obtained by the shallow network are retained. And more details are recovered during upsampling process of the decoder. From the segmentation results, it can be seen that these networks are more accurate in segmenting the details of brain tumor than Deeplabv3+. The proposed method has advantages in the extraction of multiscale features and the segmentation of brain tumor details. However, according to the comparison of the prediction results with the GT, the proposed method still needs to improve the segmentation performance of tumor boundaries.

In this paper, the evaluation indexes such as IOU, DSC, and PPV are used to evaluate the segmentation results of each network. The evaluation index values of each network are shown in Table 1. It can be seen from the table that the U-Net is more effective for the segmentation of brain tumors, and the DSC values in the segmentation of the ET and the TC have reached 0.9. Both ResUNet and DenseUNet are improved on the U-Net structure, and the DSC values of the ET and the TC are improved compared with U-Net. The segmentation performance of DeepLabv3+ on brain tumor image is the worst among these networks. It can be seen from the segmentation results that the segmentation of brain tumor details by DeepLabv3+ is not accurate enough. Compared with the other four networks, the proposed method in this paper improves the feature extraction modules on the basis of U-Net and proposes the inception module and A-inception module, which is beneficial to extract multi-scale features. At the same time, the multiresolution fusion module is proposed, which effectively utilizes the spatial context information and improves the segmentation accuracy. The results obtained by the proposed method in each evaluation index are the best, and the network performance is improved.

## 5. Conclusion

This paper proposes a multiresolution fusion network model based on improved U-Net, which is used for the fine and automatic segmentation of brain tumors. The original convolution modules in U-Net are replaced by the inception modules and A-inception modules with atrous convolutions, which increases the width of the network and makes the network more conducive to the extraction of multiscale features. At the same time, multiresolution fusion modules are used between the encoder and the decoder, and more spatial details are used to segment the details of brain tumors in the decoding stage. The proposed method is compared with four networks such as U-Net, ResUNet, DenseUNet, and DeepLabv3 +. The evaluation index values of the proposed method are better than other methods in WT, TC, and ET, and the best segmentation performance is obtained. However, the proposed method still lacks in the segmentation of some brain tumor boundaries. In the future, we will continue to improve the accuracy of the boundary segmentation of the network.

## Figures and Tables

**Figure 1:** The structure of inception module.

**Figure 2:** The structure of A-inception module.

**Figure 3:** The structure of multiresolution fusion module.

**Figure 4:** Overall architecture of the MRF-IUNet model.

**Figure 5:** The structure of ASPP module.

**Figure 6:** Example segmentation results on the BRATS dataset. From left to right and top to bottom are the segmentation results of U-Net, ResUNet, DenseUNet, DeepLabv3 +, MRF-IUNet (proposed), and ground truth. The whole tumor (WT) class includes all visible labels (a union of green, yellow, and red labels), the tumor core (TC) class is a union of red and yellow, and the enhancing tumor core (ET) class is shown in yellow.

**Table 1:** Segmentation performance of different models.

Model	DSC			IOU			PPV		
	ET	WT	TC	ET	WT	TC	ET	WT	TC
U-Net	0.9222	0.7696	0.9004	0.8998	0.7412	0.8805	0.9371	0.7828	0.9106
ResU-Net	0.9332	0.8167	0.9123	0.9107	0.7893	0.8915	0.9493	0.8373	0.9208
DenseU-Net	0.9339	0.7336	0.9225	0.9124	0.7057	0.9042	0.9526	0.7444	0.9356
DeepLabv3+	0.8986	0.6819	0.8745	0.8697	0.6504	0.8521	0.9215	0.6922	0.8839
MRF-IUNet	**0.9410**	**0.8329**	**0.9324**	**0.9195**	**0.8049**	**0.9137**	**0.9560**	**0.8489**	**0.9419**

## Data Availability

The data used to support the findings of this study are available from the corresponding author upon request.
